RETRACTED

# Fungal- and Algal-Derived Synthesis of Various Nanoparticles and Their Applications

**DOI:** 10.1155/2022/3142674

**Published:** 2022-09-26

**Authors:** Anugrah Michael, Aniket Singh, Arpita Roy, Md. Rabiul Islam

**Affiliations:** ^1^Department of Biotechnology, School of Engineering & Technology, Sharda University, Greater Noida, India; ^2^Department of Pharmacy, University of Asia Pacific, Dhaka, Bangladesh

## Abstract

Nanoparticles synthesis through biological mediated methods with a particular focus on the processes mediated by fungi and algae is discussed, which systematically reviews nanoparticle characterization, composition, synthesis methods, and, lastly but not least, the applications of NPs across five different categories to provide a reference for future research. Most traditional methods to generate nanoparticles have certain limitations, like the toxicity of precursor materials, the need for high-temperature management, and the high cost of synthesis, which ultimately hinders their utility in sectors. Greener synthesis through fungus and algae done through bioreduction by biomolecules or enzymes present in them is low-energy, low-cost, and needs a low-temperature environment, providing a unique technique for the manufacture of various metallic nanoparticles utilized in an array of industries and healthcare.

## 1. Introduction

Nanotechnology is a recent area that is rapidly growing in popularity. It involves the creation, modification, and application of materials with sizes in the range of a few micrometers to individual atoms [1–3]. Richard Feynman's through his landmark lecture, “There's Plenty of Room at the Bottom,” in 1959, provided the scientific world with a rational way to miniaturize and develop current technologies [4]. Conventional light microscopy has a limit of resolution. For simple microscopy, it is 0.4–0.7 micrometers and for compound microscopy, it is up to 200 nm. Therefore, to observe such very minute particles, a need for unique analytical tools is required because the wavelength of visible light is between 400 and 700 nm, which can cause diffraction and other optical phenomena making it difficult to observe [5].

Nanoparticles are created by a range of physical, chemical, and biological methods, of which some are new and others are some are relatively typical [1]. NPs have distinct physicochemical, structural, and morphological properties that are significant to broad-scale applications in the electronic, optoelectronic, optical, electrochemical, environmental, and biological domains, depending on their origin and synthesis techniques (Figure 1). With revolutionary methods for illness treatment and quick disease diagnosis, nanobiotechnology possesses a latent ability to revitalize the health sector, medicine, agriculture, and the food sector. As a result, effective bioassisted nanoparticle manufacturing and uses should be found, as well as their behavior and accumulation inside animals and plants [7].

RETRACTED

Living organisms have an enormous dormant capacity for producing nanoparticles possessing many opportunities for use [1]. For the generation of nanoparticles, biosynthetic approaches use microorganism cells or plant extract. Both Ag and AuNPs were synthesized through greener methods. The reaction took place at room temperature. Some microorganisms, such as bacteria, fungi, and especially yeast, are utilized to produce nanomaterials among biological species that produce nanoparticles [8]. The mechanisms behind the generation of NPs by biological organisms must be understood to build more reliable and repeatable biosynthetic methods [9]. Compared to their large-size counterparts, they have diverse qualities depending on their size, shape, charge, and surface area [10–12]. These distinct characteristics are even being used to combat several infectious disorders that are believed to be linked to dangerous bacteria. Nanoparticles have a quicker time entering pathogenic cells and interfere with cellular contents by binding protein and DN, causing apoptosis only due to their small size and surface charge. From time to time, the antibacterial activity of NP has been investigated through a range of microorganisms, including viruses, bacteria, and fungi [13].

## 2. Characterization of Nanoparticles

The generation of NPs with various chemical compositions, sizes, and regulated monodispersity is an essential topic of nanoparticle study [9]. To characterize the nanoparticle's morphology, analytical methods such as *X*-ray powder diffraction (XPD), UV-visible spectroscopy (UV-Vis), transmission electron microscopy, scanning electron microscopy, and zeta potential studies were used [8].

### 2.1. Size and Surface Morphology

To measure particle and cluster size of nanoparticles, microscopic techniques like Transmission Electron Microscope (TEM) and Scanning Electron Microscope (SEM) are used. In addition to this, photon correlation spectroscopy and gaseous Scanning Mobility Particle Sizer (SMPS) are adopted, providing faster precise measures than other methods. To measure samples in solid and liquid phases laser diffraction method is also quite popular in use [12, 14].

The shapes and surface morphology of NPs play a significant importance in utilizing their characteristics; tubular, cylindrical, conical, spherical, flat, and irregular forms with crystalline or amorphous surfaces with uniform or imperfections on the surface are some examples [15].

RETRACTED

Electron microscopy methods are a key to determining the shape of polymeric nanoparticles and other objects whose toxicity may be determined by their form [16].

*Phoma glomerata* was shown to produce silver nanoparticles (SNPs) outside of the cell. According to Gade et al., the shape and size of the mycofabricated SNPs were determined by TEM [17]. Philips CM200 super twin TEM, which operates at 200 kV (0.23 nm resolution), was used to take TEM micrographs. Another most effective approach for studying nanomaterials is *X*-ray diffraction analysis. It gives information on nanomaterial structure, peak intensity, location, and breadth [18].

### 2.2. Composition

There are several instances where the efficiency of nanoparticles was reduced due to the presence of secondary or unwanted components, as the amount of these components increased in the secondary reactions of nanoparticles and the overall manufacturing process was hampered [19].

*X*-ray photoelectron spectroscopy (XPS) or mass spectrometry, atomic emission spectroscopy, and ion chromatography are widely used methods for determining composition. The stimulation of the surface plasmon resonance band in the UV-vis range gives silver nanoparticles a yellowish-brown hue in an aqueous solution. A narrow plasmon absorption band visible in the 350–600 nm range is the most distinguishing feature of the silver sol.

### 2.3. Surface Charge

The charge on the surface of the nanoparticle regulates how it interacts with its target. A zeta potentiometer is frequently used to assess the surface charge and predict its stability in solution. Using Zetasizer Nano ZS, IONPs are synthesized using *Penicillium* spp. They noticed that the zeta potential impacted the stability of IONPs (Malvern, UK). The zeta potential voltages are in the range of 200 to +200 mV. Stability is indicated by a high zeta potential value (positive or negative). The charge on the surface of a nanoparticle attracts a narrow layer of ions having a charge opposite to that on the nanoparticle surface. This analysis used traditional analytical approaches such as UV spectroscopy, liquid chromatography (HL) after ultracentrifugation, gel filtration, or centrifugal ultrafiltration [20].

### 2.4. Crystallography

It refers to the science of distributing atoms and molecules and how they are arranged in a crystal solid. The structural organization of NPs was obtained by using powder *X*-ray, electron, or neutron diffraction techniques [19]. The *X*-ray diffractometer can also tell you about crystal structures and phases [17].

## 3. Types of Nanomaterials

Organic (liposomes and polymers), inorganic (metals, metal oxides, ceramics, and quantum dots), and carbon-based (graphene, fullerenes, and nanotubes) nanoparticles are the three broad types of NPs [21, 22].

RETRACTED

### 3.1. Organic Nanoparticles

Organic nanoparticles are frequently employed in biomedical fields, such as medication delivery systems, since they are effective and may be injected into particular regions of the body, a process known as targeted drug delivery [19]. Proteins, peptides, and lipids make up organic nanoparticles. Nanomaterials such as dendrimers, liposomes, protein or lipid-based nanomaterials, and micelles fall within this category [23].

### 3.2. Liposomes

Nanoliposomes are liposomes with vesicles within nanoscale size. Liposomes can arise in a variety of sizes, ranging from 15 nm to several nanometers, and can have a single layer (unilamellar) or several phospholipid bilayer membranes (multilamellar) [24]. They are spherical in form, with a membrane bilayer made up of amphiphilic lipid molecules. Their qualities and structures dictate how they are used in a process, particularly in medical settings [25]. Liposomes are used primarily in cancer therapy to administer chemotherapeutic medications but are also widely used in the delivery systems of a variety of anticancer treatments to improve efficacy. They can also include various bioactive components, such as medicinal medications or food additives. Because of their excellent biocompatibility and biodegradability, liposomes have a lot of promise in nanomedicine, as well as in the food and cosmetics sectors. Nanoliposome technology has advanced significantly in recent years, providing substantial prospects for food technologists in areas such as controlled release and encapsulation of food components, as well as improved stability and bioavailability of sensitive substances [21].

### 3.3. Polymeric Nanoparticles

For decades, polymeric nanoparticles have been manufactured to be utilized in a range of high-performance materials such as high-impact polymers and specialty coatings [24]. Polylactic-co-glycolic acid (PLGA), polyglycolic acid (PGA), and polylactic acid (PLA) are among the extremely biocompatible polymers used. They have a lot of surface modification potential and an excellent pharmacokinetic profile as its solubility size and could regulate throughout the process of manufacturing and are therefore used for drug delivery approach [21].

### 3.4. Inorganic Nanoparticles

Inorganic nanoparticles are safer than organic nanoparticles because they are nonbiodegradable and biocompatible and have minimal cytotoxicity. Because they have distinct optical and electrical qualities, they may be readily molded into numerous shapes during manufacture. Various inorganic constituents such as silica (SiO_2_), iron (Fe), magnesium (Mg), gold (Au), silver (Ag), graphene, and oxides are included in this category [23].

RETRACTED

Metal nanoparticles have piqued the fascination of scientists over centuries, and they may now be broadly used across biological and engineering fields. These particles can now be generated and modified with various chemical useful corporations, allowing them to conjugate with ligands, antibodies, and drugs of choice, starting a humongous variety of prime applications in magnetic separation, centered drug shipping, biotechnology, and motors for gene and drug transport, in addition, used in medical diagnostics. Silver nanoparticles are displaying promise as cancer treatment [26].

The iron oxide nanoparticles are stable and have a near-neutral zeta potential. They are also large enough to escape renal clearance. Metal oxide nanoparticles have superparamagnetic, which is an essential feature because it makes MRI contrast agents to target SPIONs [26].

### 3.5. Carbon-Based Nanoparticles

Due to their low toxicity and biological compatibility, carbon-based N such as graphene oxide, fullerenes, nanodiamond, graphite, and others have been widely implemented and used in biomedical applications (diagnostics and therapies) [23].

They are dielectric, semiconducting, conducting, and superconducting and can be employed as structural and electrical materials [5].

In recent years, graphene's outstanding properties, including optical property, high thermal conductivity, high current density, chemical stability, ballistic transport, and prime hydrophobicity, have piqued attention as a multi-functional material. Because of its unusual electrical properties, graphene has been employed in electronics applications such as transistors, transparent conducting electrodes, field emitters, integrated circuit modules, electrochemical and biosensors [27].

A fullerene is a molecule with 60 carbon atoms that takes the shape of a hollow spherical, ellipsoid, or tube. Buck balls are spherical fullerenes, while carbon nanotubes or buck tubes are cylindrical fullerenes. Fullerenes have a graphite-like structure, made of stacked grapheme sheets with connected hexagonal rings, but they can also have pentagonal (or even heptagonal) rings, resulting in potentially porous molecules. Endohedral fullerenes are made of buckyball clusters or buck balls with less than 300 carbon atoms and include the most common fullerene, buckminsterfullerene, and C60 [24].

Carbon nanotubes are nanostructures structured of rolling graphene planes that have a ton of physicochemical characteristics and have wide applications in the biomedical field. The discovery of carbon nanotubes using high-resolution electron microscopy (HREM) has sparked a flurry of experimental and theoretical research on the material [26].

RETRACTED

Nanotubes are carbon-based long thin tubular materials formed from carbon crystals, diamonds, or unbreakable hexagonal graphite layers in a concentric way [23].

## 4. Methods

Because of their extraordinary capabilities, regulated by its structural morphology, NPs have been intensively researched, and numerous studies have employed in chemical and physical approaches to synthesize nanoparticles [28].

The commercialization of high-throughput NPs with acceptable and regulated quality is needed in a variety of sectors. To make NPs, two traditional methods are routinely used. Both techniques have different synthesis principles but yield NPs with the required properties. Nanoparticles are made using a variety of processes that can be classified as a top-down or bottom-up method [18].

### 4.1. Top-Down Method

The bulk materials were compressed bit by bit in the top-down technique, resulting in fine generations of NPs [29]. Lithography, sputtering, and mechanical techniques such as thermal evaporation, milling and grinding, chemical etching and photo reduction are used to accomplish this [30]. Major merits, which set them apart for nanoparticle synthesis, include production cost, control over size, and morphology, ensuring overall dimensional stability of the final product and a monodisperse population of higher production enabling industrial level bulk production. Furthermore, they increase drug stability and encapsulation efficiency [31].

This method is suitable for generating materials and making particle-to-particle connections and is the rational method for the production of Ns in large numbers. On the other hand, disadvantages include NPs surface imperfection and particles could take damage [32]. Due to the physiochemical characteristics of Ns being relative to surface design, the top-down method for N synthesis is limited to particular applications.

### 4.2. Physical Methods

They include creating Ns using material abrasion, melting, and evaporation using mechanical pressure, high-energy radiations, thermal energy, or electrical energy. These techniques primarily use a top-down approach and are preferred because they are solvent-free and create uniform monodisperse NPs. High-energy ball milling, laser ablation, electrospraying, inert gas condensation, physical vapor deposition, laser pyrolysis, flash spray pyrolysis, and melt mixing are some of the most frequently utilized physical ways to create. On the other hand, physical procedures are less cost-effective because of the large amount of waste created during the synthesis. Physical procedures require a large amount of energy. To create nanoparticles, physical and photochemical processes need extremely high temperatures, vacuum conditions, and expensive equipment.

RETRACTED

### 4.3. Bottom-Up Method

There are various methods that are included in the bottom-up technique, which include processes such as metal ion chemical reduction or oxidation, solid-gel chemistry, coprecipitation, microemulsion, chemical vapour deposition, hydrothermal, pyrolysis, radiation driven, solvothermal, and electrodeposition procedure, also called wet chemical processes. Self-assembly, or bottom-up synthesis, entails assembling nanoparticles from small components such as molecules, atoms, and smaller particles. However, the use of potentially dangerous and harmful substances, higher costs, toxicity, high concentrations of consumption levels, and long recovery time and wastage have harmed them.

#### 4.3.1. Chemical Method

Various chemical methods for making nanoparticles are proposed, and the majority are now routinely employed to create nanostructured materials [33]. The following are some of the most frequently used chemical processes for producing NPs: polyol synthesis, chemical vapor synthesis, the sol-gel method, microemulsion, hydrothermal technique, and plasma accelerated chemical vapor deposition method. The majority of chemical procedures involve hazardous reducing agents, including sodium citrate, ethylene glycol, and sodium borohydride; however, they produce poor particle sizes and no control oversize distribution.

The high cost of this synthetic approach and the hazardous properties of this synthetic approach may limit its usage on a large scale. Furthermore, the items created using this method are inefficient [34].

#### 4.3.2. Biological Method

Greener nanotechnology to reduce the ill impacts of nanomaterial fabrication is the optimum method as it lowers the chances of difficulties that come with other approaches [27]. To synthesize and produce NPs, biosynthesis, also called greener synthesis, offers an environment-friendly, less toxic, low-cost, and rational method. The bottom-up method for NP synthesis is biological synthesis. The formation of nanoparticles using biological methods requires the participation of various biological agents such as viruses, bacteria, fungi, algae, and plants. But care should be taken that these fungi and viruses or bacteria utilized in NP generation should not cause any problem and when getting in contact with the human body, they should be nonpathogenic in nature [2, 35].

Green synthesis is a process including metals in its atomic form clustering with each other and then forming nanoparticles; it is made using the bottom-up method. Reduction through biomolecules is connected to the greener concept; except instead of expensive and harmful chemicals, green materials are employed to produce nanoparticles. Researchers developed adverse reaction monitoring to discriminate between reduction of nanoparticles using greener methods and typical wet chemistry approach. [36].

RETRACTED

Green nanoparticles had considerably lower cytotoxicity and phytotoxicity than wet chemical nanoparticles, suggesting that they are safer for use in research related to melanoma treatment [37].

As a result of its ecologically friendly nature, it is the best technique or gives the best outcomes among fundamental green chemistry approaches. The structure and morphology of generated NPs are greatly influenced by the organism's nature. An incredible variety of nanoparticles with various forms and sizes resulted from an array of biological organisms.

Through a brown algae *Cystoseira baccata*, AuNPs are produced, which offer tremendous promise in the treatment of colorectal cancer. Similarly, fungus like *Neurospora crassa* and *Fusarium oxysporum* are subjects of interest for the feasible “scale-up” option for PtNP production [38].

Three types of bioassisted nanoparticle synthesis technologies may be distinguished: (i) microorganism-based biogenic synthesis; (ii) plant extract-based biogenic synthesis; (iii) fungal drive nanoparticles; (iv) algal drive nanoparticles.

*(1) Plant Extract-Based Nanoparticles Synthesis.* Plants extracts and biomass has become a good way to synthesize nanoparticles as their manufacturing is more efficient, they are easy to make compared to chemically manufactured NPs, and they are nontoxic, making them ecofriendly [12, 39, 40]. Metal-based NPs are the main focus of this method including metal oxide, alloys, and inert metals; this is possible due to the presence of a wide variety of plant metabolites that help in their creation. These metabolites act as reducing agents and capping agents [14, 41].

*(2) Microorganisms-Based Nanoparticle Synthesis.* Bioreactors for the production of NP include prokaryotic bacteria, actinomycetes, fungi, algae, and yeast. Huge scientific efforts went into developing this approach for creating a wide range of NPs (Pd, TiO2, Ag, Au, CdS, etc.). Microorganisms collect ions from their surroundings and use enzymes produced by cellular processes to convert metal ions into their elemental form. It might be classed as intracellular or extracellular, depending on where the NP is synthesized. Metal ions are transported inside the microbial cell to generate NPs in the presence of enzymes in the intracellular approach. In the case of extracellular NP production, the metal ions are trapped on the cell surface and ions get reduced in the presence of certain enzymes [42].

RETRACTED

Compared to plants and bacteria, fungi and algae are excellent sources for nanoparticle manufacturing. Algae and fungus are easy to cultivate and produce a large quantity of biomass in a short amount of time, making them a suitable source for NP synthesis [32]. Fungi also have a remarkable capacity to synthesize various bioactive chemicals with uses in various fields. Their form and size can be adjusted and are commonly used as reducing and stabilizing agents. Algae may also be used in manufacturing a variety of bioactive chemicals, pigments, and proteins that aid in salt reduction and serve as capping agents in the production mechanism.

## 5. Fungi-Based Synthesis

Fungi can be used to produce nanoparticles with well-defined dimensions. According to research, fungus, as opposed to bacteria, might be a source for large-scale nanoparticle synthesis. Fungi are known to secrete many more proteins and chemicals than other organisms; as a result, in a biosynthetic method, the productivity of nanoparticles could be considerably increased [1]. Specialized enzymes released by fungi, such as reductases, bring up the intriguing prospect of constructing a rational biosynthesis method for nanomaterials with various chemical compositions [43].

Using fungal and actinomycete-mediated green chemistry to synthesize nanoparticles offers several benefits, including ease of scaling up, economic feasibility, and the potential to cover huge surface areas quickly with appropriate mycelia development. The switch from bacteria to fungus to create a natural “nanofactory” provided the benefit of significantly simplifying the downstream processing and handling of biomass [44] (Figure 2).

Two methods are utilized to produce fungi-mediated nanoparticles: intercellular and extracellular processes.

### 5.1. Intracellular Synthesis

When a metal precursor is given to a fungal culture, the precursor is internalized by the biomass. Because NPs are trapped within, extraction operations such as centrifugation, filtering, and other methods are necessary to liberate them [1,45].

*Verticillium* sp., an acidophilic fungus, was isolated from a *Taxus* plant and treated to AgNO_3_, resulting in creating Ag nanoparticles.

Gold (Au) and silver (Ag) nanoparticles have extraordinary colors caused by the activation of surface plasmon vibrations in the particles (pink to blue for gold and light yellow to brown for silver), and thus, they give an easy way to visually determine their existence inside biomass of fungi. Silver nanoparticles are generated just within the biomass, not outside of it, which is an intriguing aspect of this specific fungus [44].

RETRACTED

Mukherjee et al. used the fungus *Verticillium* to develop a fungal-assisted biological technique for synthesizing silver NPs. When fungal biomass is exposed to aqueous Ag+ ions, it is reduced intracellularly to silver NPs with a diameter of 25 12 nm. Microscopic examination reveals that the surface of the mycelia is the primary location for the production of NPs, catalyzed through enzymes found in the mycelia cell wall [46].

### 5.2. Extracellular Synthesis

Extracellular enzyme secretion has the benefit of getting large numbers in a reasonably pure condition, devoid of external biomolecules like protein associated with the organism, and therefore could be simply handled through ultrafiltering cells and separating the enzyme for nanoparticle creation from the cell-free filtrate [44].

To the aqueous filtrate containing fungal macromolecules, a metal precursor is introduced. The process is widely used since it does not require any additional techniques to release NPs from the cell [9].

The proteins and reducing agents released by fungus stabilized extracellularly generated nanoparticles. In connection with nanoparticles, it has been found that fungal biomass contains four high mass proteins. The strain-specific NADH-dependent reductase was one of them [1].

In a study, *Cladosporium cladosporioides* fungus was used to perform extracellular production of silver nanoparticles (AgNP). TEM scans show that the AgNP was of size 10–100 nm. *Penicillium fellutanum*, isolated from coastal mangrove soil, accomplished the production of silver nanomaterials in vitro using AgNO3 as a precursor in 2009 [47]. When the culture filtrate was treated with 1.0 mmol L–1 AgNO3, kept at 0.3 percent NaCl and pH 6.0, and incubated at 5°C for 24 hours, the biogenesis of the nanoparticles reached its peak. Filamentous fungi are a promising possibility for metal nanoparticle production. As a result, Bhainsa et al. used the filamentous fungus *Aspergillus fumigatus* to examine the production of AgNPs extracellularly [48].

To summarize the process of extracellular synthesis, various steps are followed that are given below [9, 17, 44, 49]:

1. Culture fungus on agar or any other nutrient medium
2. Production of biomass
3. Transfer to liquid medium
4. Filtration is required and biomass is discarded
5. Silver nitrate solution (AgNO_3_) added to the filtrate [Ag+ and NO_3_−]
6. Reduction of Ag+ to Ag° by fungal biomolecules (Ag° is the elemental form)

On a nanometric scale, enzymes found in fungal filtrate convert silver ions to elemental silver. When this happens, the color of the filtrate changes, which may be seen using UV spectroscopy. The main enzymes responsible for reducing the silver ion are NDH-dependent nitrate reductase and NDH. The synthesis of different nanoparticles from different fungal species has been summarized in Table 1.

RETRACTED

## 6. Algae-Derived Synthesis

Algae are photosynthetic aquatic filamentous creatures that belong to the domain Plantae. They may be unicellular or multicellular creatures, are omnipresent, and live in freshwater, seawater, and the surface of damp rocks. They are important in medical, pharmaceutical, agricultural, aquaculture, and cosmetics. Microalgae and macroalgae are the major forms of algae. Microalgae must be observed with a microscope, but macroalgae may be counted with the naked eye. Algae are also commonly used to tackle the negative drawbacks of chemical or physical treatments. No additional reagents are required, as the cell wall of the alga contains functional groups and biomolecules that serve as reducing agents [64]. Algae are frequently referred to as bionanofactors, since they can produce nanoparticles from both live and dead material (Figure 2). Chlorophyceae, Phaeophyceae, Cyanophyceae, Rhodophyceae, and various species of diatoms are the algae that are the most commonly used for metallic nanoparticle manufacturing. Compared to the wet chemical approach, algae can decrease metal ions that build inside them, they are easier to handle, and the residuals created during synthesis are less hazardous and pose less of a threat to the environment. Additionally, the total process is energy-efficient. Algae can collect metals and decrease metal ions, have less temperature modifications, can tremendously lower energy expenditure, and, last but not least, are less toxic, proclaiming that they are the best alternative for NPs synthesis [65].

The production NPs through algae is faster than the synthesis of nanoparticles using any other bioagents [18]. In contrast to most biomass, micro- and macroalgae may be harvested anytime in a single year. Algae may also develop without the need for any external chemicals or fertilizers. Microalgae develop at a breakneck pace, doubling their bulk ten times quicker than higher plants [66]. The algae extract is made by boiling or heating algae in an organic solvent or water for a set amount of time, which results in the synthesis of nanoparticles. Then ionic metal compound molar solutions are created. Finally, the ionic metal compound molar solutions and the algal extract solution are combined and incubated for a set amount of time under regulated culture conditions with continuous mixing or without mixing.

RETRACTED

The steps involved in the synthesis of algal nanoparticles are as follows:

1. Culture the algae and transfer it to water/solvent by boiling it.
2. Prepare the ionic solution of the metallic compound in molar terms.
3. Incubate and mix the algal extract with a metal compound solution with constant stirring.
4. Color change in the solution is observed.

The synthesis of different nanoparticles from different algal species has been summarized in Table 2.

## 7. Applications

### 7.1. Antibacterial and Antifungal Activity

Antibiotic resistance is a global challenge to science; consequently, it is critical to producing a significant innovative material to combat antimicrobial-resistant strains. As a result, scientists engineered nanometal or metal oxide NPs to generate antibacterial activity. Metallic NPs were shown to have a humongous array of biocidal properties against Gram-positive bacteria, Gram-negative bacteria, and eukaryotes [92]. The antibacterial activity of ZnO NPs against test bacteria is affected by surface area, shape, particle size, and other factors [93]. To achieve maximum antibacterial action, tiny nanoparticles must be produced, and their size must be kept practically constant. The ZnO NPs produced by the fungus were pure, mostly hexagon-shaped, belonging to size 34–55 nm. Inhibition of Gram-negative and Gram-positive bacteria was effectively observed by the biosynthesized ZnO NPs. The antifungal efficacy of ZnONPs produced from fungi was relative to the dosage. Different doses inhibited *E. coli*, *B. cereus*, *S. aureus*, and *P. aeruginosa*, corresponding to significant differences in sensitivity to ZnO NPs. The antibacterial activity of fungal-synthesized ZnO NPs was dose-dependent, and as particle concentration increases, antibacterial activity also increases [60].

In addition, smaller AgNPs had better antibacterial activities against *E. coli* and *S. aureus*. Nanoparticles smaller than 10 nm have been proven under several investigations to reach the inside of bacterial cells, increasing their bactericidal activity [61]. Finally, antibiotic ampicillin and econazole nitrate demonstrated greater antibacterial activity against bacteria and mold, respectively, when compared to AgNPs. This suggests that standard antibiotics retain their antibacterial effectiveness [61]. Antibacterial properties of iron oxide NP generated from the genus *Penicillium* using the disc diffusion method. They were tested at different concentrations of 100 g to 250 g. *S. sonnei* (ATCC 25931), *S. aureus* (ATCC 33862), *P. aeruginosa* (ATCC 15442), *E. coli* (ATCC 25922), and *K. pneumonia* (ATCC 13883) were the bacteria used in this work [20].

RETRACTED

The antibacterial action of NPs produced by algae is well recognized. *Bifurcaria bifurcate*, brown algae used to isolate copper oxide nanoparticles ranging 5–45 nm with antibacterial activity against *Enterobacter aerogenes* (Gram-negative) and *S. aureus* (Gram-positive) [94]. An aqueous extract of diatom, Amphora46, was used in a recent report on the photoinduced generation of polycrystalline AgNP using fucoxanthin, a photosynthetic pigment involved in reducing Ag+ ions. Additionally, the antibacterial activity of AgNP produced against Gram-positive and Gram-negative bacteria was evaluated [69]. Antifungal compounds made from algal NPs were shown to be effective. Only a small amount of work has been done in this area. Marimuthu et al. showed an antifungal effect against *Humicola insolens*, *Fusarium dimerum, Mucor indicus*, and *Trichoderma reesei* through an aqueous extract of red algae, *Gelidiella acerosa,* as a reducing agent [94].

### 7.2. Anticancer Therapy

Cancer is a terrible global illness that causes substantial health issues and mortality, with 8.8 million people dying from it in 2015. Since they possess increased surface area, biological NPs are a burgeoning sector in cancer therapy, allowing for efficient drug administration, tumor selectivity, and promising action. To improve anticancer treatment, it is now essential to conduct research using in vivo models to expand in vitro studies and to specify biological parameters [92]. Boca et al. [95] reported a chitosan-coated silver nanotriangle was produced as a photothermal agent for a panel of human non-small-cell lung cancer cells (NCIH460) [95]. Similarly, *Sargassum vulgare* was used to prepare silver nanoparticles of 10 nm in size and understand its ability to target malignant human myeloblastic leukemia cells HL60 and cervical cancer cells HeLa [96]. The fungus *asparaginase* was used to generate gold nanoparticles highly suitable for targeted drug delivery for cancer management [97]. The cytotoxicity of nanobiocomposites was reported to be greater against lung cancer cell line A549 than against ovarian cancer cell line A2780. The asparaginase gold nanobiocomposite, which was created, can be used as an effective anticancer drug with enhanced bioavailability against the lung cancer cell line A549, which has a toxicity range of 84.5 percent. For the past decade, nanoparticles derived through microalgae have been utilized in drug delivery. Compared to other carriers, these have less toxic properties, biodegradability, and a larger surface area. Microalgae are used to produce antibodies, vaccines, growth factors, and certain hormones required in medical biotechnology [98, 99].

RETRACTED

Targeted delivery of drugs or genes to tumor cells is achieved through a drug delivery system. Generally, due to mutation, many genes are miscoded or absent in people with genetic disorders. Therefore, using silica nanoparticles as gene taxi is thought to be fruitful [100]. Because they transport pharmaceuticals, ingenious drug delivery can overwhelm the impediments of conventional methods of medications, such as low stability and high toxicity. Some of the most commonly utilized drug carriers are micelles, liposomes, and silicon oxide NPs, each with its own set of benefits and drawbacks. Silica-based nanomaterials, such as MCM-41 and SBA-15, exhibit wide surface area, customizable pore size, high loading capacity, and thermostability. Their synthesis was found to be costly and time-consuming, as well as requiring high energy and hazardous ingredients.

### 7.3. Bioremediation

Heavy metals are nonbiodegradable, have health hazards, and cause ill effects on the ecosystem. They cause mutagenesis, cancer, and inherited genetic problems by binding to the same locations as necessary metal ions and causing structural and biomolecular instability. Traditional techniques for removing heavy metals are well-established but have numerous limitations. As a result, additional ways to effectively remove heavy metals are required. Nanoparticles have a lot of promise and are employed as adsorbents to remove heavy metals from water bodies due to their maximum adsorption and high selectivity [11]. Through dead fungal biomass, the isolation of extracellular copper nanoparticles is a cheaper and greener approach that may also be used for the bioremediation of damaged areas. First, the fungus *T. koningiopsis* explored the possibility of removing copper ions and reducing them to copper NPs, expanding the range of organisms to synthesize metal nanoparticles for biological wastewater treatment. Fungal-mediated biosynthesis of copper NP appears to be a potential technique for expanding industries and technical copper NPs production as it seems to be a viable candidate [9]. NP procurement as a new strategy to remediate polluted environments has recently gained much attention. Algal-derived nanoparticles are used as bioremediation agents; for example, AgNPs isolated from *U. lactuca* photocatalyze methyl orange dye degradation. Furthermore, even a low concentration of these nanoparticles was found to significantly reduce the growth of *Plasmodium falciparum*, which is a chloroquine-resistant parasite [101]. Compared to cyanobacterial extract, AgNPs produced from Microchaete demonstrated superior decolorization activity against methyl red azo dyes [102]. AuNPs produced from the aqueous extract of brown algae *S. tenerrimum* and *T. conoides* were shown to have catalytic activity against the organic dyes sulforhodamine, rhodamine B, and aromatic nitro compounds in another work [103].

RETRACTED

### 7.4. Larvicidal Activity of Nanoparticles

Vectors are carriers of certain disease-causing substances such as mosquitoes, mites, and fleas. Vector-borne diseases account for more than 17% of all attractive infections, killing more than 700,000 people annually. Dengue fever is a well-known viral disease transmitted through *Aedes aegypti*. Other vector-mediated viral diseases include chikungunya fever, decavirus fever, yellow fever, West Nile fever, *Japanese encephalitis* (all mosquito-borne), and tick-borne encephalitis [92]. The efficiency of mycogenic silver nanoparticles (AgNPs) generated from *Fusarium pallidoroseum* biomass was examined against a potent sugarcane pest in western Uttar Pradesh, which is called white grubs, *Holotrichia serrata*. In vitro, the AgNPs were given to third instar white grub larvae, and the fatal dosage (LD50) was calculated using Probit analysis, which was then confirmed and determined to be significant at the 0.05 level using the chi-square test [104]. *Sargassum myriocystum*, a marine natural resource seaweed, was employed in this study because of its distinct phytochemicals and major features in providing excellent responses to numerous biological applications. It mediates titanium oxide nanoparticles to be a strong disrupting substance for bacteria and larvae of mosquitoes [105].

### 7.5. Biosensors

Biosensors are now widespread in biomedical diagnostics and many other areas such as tracking disease progression, environmental monitoring, drug discovery, and forensics. A variety of technologies can be used to develop biosensors. By binding to high-affinity biomolecules, many analysts can be detected with high sensitivity and selectively. Biosensing applications can be investigated using NPs generated by algae. AuNPs, for example, have been shown to be a useful technique for detecting hormone (hCG) for the pregnancy test [106]. To remedy allergies, coronary heart attacks, cardiac operations, and asthma, platinum NPs function as a brand-new biosensor corresponding to brilliant sensitivity for the detection of adrenaline. Algae-derived AuNP has excellent optical properties that are useful for determining the type and number of hormones in our body, which is an important aid in diagnosing cancer. Micro-AuAg alloys synthesized from algae at ambient temperature show significant electrocatalytic potential for 2-butanone and can detect initial cancer cells [107, 108]. Through a recent study, AgNP mediated by *Noctiluca scintillans* was tested for the detection of colorimetric hydrogen peroxide (H_2_O_2_). It is a disinfectant that helps with small abrasions, tooth discomfort, whitening teeth, and mouth drainage. The results revealed that degradation of hydrogen peroxide on AgNP's catalytic surface was temperature-, duration-, and pH-dependent. This test likewise revealed a color shift from brown to colorless, exhibiting the most dramatic color shift [109]. In another investigation, AuNPs produced by *Hypnea valencia* were shown to be capable of detecting human chorionic gonadotropin hormone levels from urine samples from pregnant women [106].

RETRACTED

## 8. Future Prospects

Nanoparticles have demonstrated significant promise in various sectors, including medicine, environmental biology, and electronics. Though, developing sustainable techniques for the synthesis of these nanomaterials remains a problem. The majority of studies to date are accomplished on a laboratory scale setup, and future progress in this area will be contingent on collaboration from industries plus a thorough evaluation of the economic and environmental implications, as well as optimization of current resources for adequate bulk production. Future research should focus on developing nanoparticles with low toxicity, low-energy consumption, and high catalytic activity and maximizing antibacterial properties. As a result, it is critical to synthesize metallic nanoparticles, particularly using biogenic synthesis methods, which are employed in various disciplines such as cancer therapy, medication transport, and biosensor development.

## 9. Conclusion

We have presented a detailed overview of current advances in the fungal- and algal-derived generation of nanoparticles in this article. This study focuses on the idea and need for producing metallic nanoparticles from diverse fungi and algae. Furthermore, in light of recent discoveries, we argued for the use of nanoparticles for antibacterial, antioxidant, anticancer, anti-inflammatory, biosensors, and larvicidal properties. Nanotechnology is a powerful field that allows applied science to control molecules at the molecular level. Both physical and chemical methods of producing nanoparticles have downsides due to the radiation and toxic substances involved. The greener synthesis of NPs is based on the premise that it should be a benign process that uses living resources, avoids toxic components, is nontoxic, and is cost-effective. Developing new “environmentally friendly” synthetic processes for producing nanostructured materials at a lower cost and with less energy might lead to a wider variety of nanotechnology applications. We believe that by employing ecological approaches, we will be able to synthesize nanomaterials with regulated properties in a short period of time for consistent NP preparation in the laboratory, and it may be developed as a safe alternative method for large-scale NP manufacturing in the near future.

RETRACTED

## Figures and Tables

**Figure 1:** Applications of nanoparticles and nanostructure [6].

**Figure 2:** Fungal and algal synthesis of nanoparticles.

**Table 1:** Fungi-derived nanoparticles.

S.No	Name of species	Metal	Size (nm)	Mode	References
1	*Verticillium* sp.	Au	20	Intracellular	[46]
2	*Fusarium oxysporum*	Au	20–40	Extracellular	[49]
3	*Schizosaccharomyces pombe* (yeast)	CdS	1–1.5	Intracellular	[50]
4	*Colletotrichum* sp.	Au	20–40	Extracellular	[51]
5	*Fusarium oxysporum*	ZrO2	7–8	Extracellular	[52]
6	*Fusarium oxysporum*	TiO2 NPs	6–13	Extracellular	[53]
7	*Fusarium oxysporum*	Silica (SiF62) and Titanium particles (TiF62)	5–15	Extracellular	[53]
8	*Aspergillus fumigatus*	Ag	5–25	Extracellular	[48]
9	*Fusarium oxysporum* and *Verticillium* sp.	Magnetite	20–50	Extracellular	[54]
10	*Hormoconis resinae* (creosote fungus)	Ag	20–80 and 10–20	Extracellular	[55]
11	*Neurospora crassa*	Pt	—	Intracellular and extracellular	[56]
12	*WA 2315*	Ag	23–105	Extracellular	[57]
13	*Cladosporium cladosporioides*	Аg	10–100	Extracellular	[47]
13	*Neurospora crassa*	Аg	11	Intercellular	[58]
14		Au	32	Intercellular	[58]
15	*Trichoderma koningiopsis*	Cu	87.5	Extracellular	[9]
16	*Phoma glomerata (MTCC-2210)*	Ag	19–65	Extracellular	[17]
17	*Penicillium notatum PTCC 5074*	Zirconium	—	Extracellular	[59]
18	*Xylaria acuta*	ZnO	*34–55*	Extracellular	[60]
19	*Aspergillus japonicus PJ01*	Ag	3.8 ± 1.1 and 9.1 ± 2.9	Extracellular	[61]
20	*Phoma* sp.	Au	10–100	Extracellular	[62]
21	*Purpureocillium lilacinum*	Ag	50	—	[63]

**Table 2:** Algae-synthesized NPs.

S. no	Name	Particle	Size (nm)	Mode	Condition	Reference
1	*Sargassum wightii*	Аu	8–12	Extraсellular		[67]
2	*Tetraselmis suecica*	Аu	∼79	—	Reduction	[68]
3	*Chlorococcum humicola*	Ag	4–16	Extracellular/intracellular		[69]
4	*Sargassum myriocystum*	Au	∼15	—	—	[70]
5	*Tetraselmis kochinensis*	Au	5–35	Intracellular	Reduction	[71]
6	*Stoechospermum marginatum*	Au	18.7–93.7	—	Reduction	[72]
7	*Rhizoclonium fontinale*	Au	∼16	Intracellular		[73]
8	*Lobophora variegata*	Ag	20–60	—	Reduction	[74]
9	*Prasiola crispa*	Au	5–25	—	Reduction	[75]
10	*Sargassum swartzii*	Аu	∼35	—	Reduction	[76]
11	*Caulerpa racemosa*	Аg	5–25	—	Reduction	[77]
12	*Padina pavonica*	Au	30–100	Extracellular	Reduction	[78]
13	*Ecklonia cava*	Ag	∼43	—	Reduction	[79]
14	*Gracilaria parvispora*	Ag	12–30	Extracellular		[80]
15	*Chlorella vulgaris*	Рd	5–20	—	Reduction	[81]
16	*Padina gymnospora*	Pd	5–50	—	Reduction	[82]
17	*Sargassum wightii*	ZrO_2_ (zirconia)	∼4.8	—	—	[83]
18	*Sargassum muticum*	Ag	21.95 ± 0.96	—	—	[84]
19	*Amphiroa fragilissima*	Ag	104.6	Extracellular	—	[85]
20	*Botryococcus braunii*	Ag	40–100	—	Reduction	[86]
21	*Gelidium corneum*	Ag	20–50	—	Reduction	[87]
22	*Chlorella sorokiniana*	Au	—	Extracellular/Intracellular	Reduction	[88]
23	*Laminaria ochroleuca*	Ag	10–20	—	Reduction	[89]
24	*Sargassum coreanum*	Ag	∼19	—	—	[90]
25	*Sargassum longifolium*	CuO	40–60	—	Reduction	[91]

RETRACTED

## Data Availability

The data used to support the findings of this study are included within the article.
